# Role of social media to improve job performance with mediating role of transactive memory capability and employee creativity

**DOI:** 10.1371/journal.pone.0307292

**Published:** 2024-07-22

**Authors:** Jingyu Fu

**Affiliations:** Department of Humanities and Communication, Xinyang Agriculture and Forestry University, Xinyang, Henan, China; University of Central Punjab, PAKISTAN

## Abstract

The increased usage of social media in organizational settings has raised questions about its effect on job performance. This study explains the interplay between social media usage, transactive memory capability, employee creativity, and job performance within the Chinese organizational context. The rationale for this study stems from the need to understand how social media usage can enhance job performance through cognitive and creative processes within teams. On the basis of earlier literature, the survey questionnaire was designed to collect data and the survey included validated scales to measure these constructs. The data is collected from 816 employees in China via online resources like social media and emails and then Structural Equation Modeling is used for empirical analysis through AMOS software. The findings show the positive impact of social media on job performance while transactive memory capability and employee creativity mediates this relationship. These findings contribute to a better understanding of how social media can be leveraged to improve job performance. Practical implications highlight the importance of fostering transactive memory capability through social media platforms, facilitating employee creativity, and ultimately, bolstering job performance. Additionally, this study underscores the need for organizations to strategically harness the potential of social media as a catalyst for innovation and knowledge sharing, thus optimizing workforce performance in the digital era.

## 1. Introduction

Job performance is the effectiveness, efficiency, and quality of an individual’s work-related activities and behaviors within an organization [1]. It encompasses the outcomes and behaviors that employees demonstrate while fulfilling their job duties and responsibilities. Job performance includes various elements like task performance, contextual performance and adaptive performance [2]. The task performance is related to the core duties and responsibilities outlined in a job description. It involves how well an employee completes the specific tasks and assignments related to their role, meeting deadlines, achieving goals, and producing desired outputs [3]. The contextual performance is extra-role behavior that contribute to the overall functioning of the organization but might not be explicitly required in the job description [4]. While adaptive performance is an ability to adapt to changes in work environment, learn new skills, handle unexpected situations, and effectively adjust to evolving job demands [5]. Effective job performance is crucial for organizational success as it impacts productivity, innovation, customer satisfaction, and overall competitiveness [6]. Organizations often seek to improve job performance through training, providing resources, setting clear expectations, and offering incentives [7]. Job performance is crucial for both organizations and individuals for several reasons. In organizations, high job performance directly translates to increased productivity and efficiency [8]. Employees who perform well can complete tasks more quickly and effectively, contributing to the overall output and success of the organization. Moreover, effective job performance leads to better financial outcomes. When employees perform their tasks well, it reduces waste, improves customer satisfaction, and can result in higher sales and profitability [9]. In addition, organizations known for high job performance tend to have better reputations. This can attract more customers, investors, and top talent, further driving organizational success. In context of individuals, high job performance is often recognized and rewarded through promotions, raises, and other career advancement opportunities [10]. Individuals who perform well are more likely to climb the career ladder. Performing well at work leads to a sense of accomplishment and fulfillment, enhancing overall job satisfaction and personal happiness. Consistently high job performance usually requires continuous learning and skill enhancement. This not only benefits the current job but also improves employability and career prospects in the future [11]. Successfully meeting job expectations can boost an individual’s self-esteem and confidence. This positive self-perception can have a ripple effect, improving performance further and contributing to personal growth [12].

There are various factors which contribute to improve the job performance of an employee within firm. Social media, transactive memory capability, and employee creativity are some important factors affecting the job performance and little focused in the earlier literature. Social media has much significance in improving job performance by facilitating communication, collaboration, and networking among professionals [8]. Social media platforms and professional networking sites like LinkedIn are extensively used in China [9]. These platforms enable professionals to connect with colleagues, industry experts, and potential collaborators. Improved networking leads to better information exchange, learning opportunities, and staying updated with industry trends, thereby enhancing job performance [13]. Social media allows for the rapid sharing of information and expertise across geographical boundaries. Within organizations, platforms like WeChat Work facilitate team collaboration, file sharing, and real-time communication, fostering efficient teamwork and knowledge dissemination [14]. This facilitates problem-solving, decision-making, and project execution, ultimately improving job performance. Moreover, these platforms often host industry-specific groups, forums, and discussions where professionals can exchange insights, best practices, and learn from each other [15]. Additionally, access to online courses, webinars, and educational resources shared through social media aids in continuous learning and skill development, contributing to enhanced job performance [13]. In China, social media is a powerful tool for professionals, fostering communication, collaboration, learning, and networking, all of which contribute significantly to improving job performance across various industries and roles [16].

Transactive Memory Capability (TMC) is an ability to collectively encode, store, and retrieve knowledge through coordination and communication among its members [17]. This concept originates from the broader theory of transactive memory systems, “which describes how groups collectively remember, store, and retrieve information” [16]. TMC allows the groups to specialize in certain domains of knowledge, recognizing others’ expertise and relying on them when needed [18]. This facilitates effective knowledge sharing and coordination, ensuring that the right information is accessible when required, ultimately enhancing decision-making and problem-solving processes [19]. When team members collaborate, this reduces redundancy in efforts, streamlines communication, and avoids errors, leading to improved task execution and productivity [20]. Groups with high TMC are more adaptable to change. As individuals rely on each other’s specialized knowledge, they can quickly adapt to new situations, learn from one another, and collectively acquire new knowledge or skills essential for addressing novel challenges or opportunities [19]. TMC fosters an environment conducive to innovation. When individuals trust their colleagues’ expertise and have easy access to diverse knowledge sources within the group, it stimulates creativity, idea generation, and the development of novel solutions to complex problems [21]. “Strategies such as cross-training, regular team meetings, knowledge-sharing platforms, and mentorship programs can significantly contribute to the development and utilization of transactive memory capability within teams and organizations” [22].

Employee creativity significantly influences job performance across various domains within an organization. Creative employees bring fresh perspectives to problem-solving [23]. They’re adept at thinking outside conventional boundaries, generating innovative solutions, and adapting to changing circumstances [24]. This ability to innovate directly impacts the efficiency and effectiveness of tasks, projects, and processes, leading to improved job performance. Employees who think creatively are more likely to embrace change, pivot when necessary, and proactively respond to new challenges [25]. This adaptability is crucial in dynamic work environments and contributes to overall job performance by ensuring tasks are completed efficiently despite changing conditions [9]. Creative individuals often consider diverse viewpoints and explore multiple alternatives before making decisions. This comprehensive decision-making process leads to more informed choices [26]. In roles related to product development, marketing, or service provision, employee creativity is instrumental. Creative input drives the development of new products, services, marketing campaigns, and strategies, contributing directly to organizational growth, competitiveness, and success [16]. Organizations can foster employee creativity by providing a supportive culture that encourages experimentation, tolerates failure as part of the learning process, offers opportunities for skill development and training, and allows autonomy in decision-making [21]. Additionally, providing resources, such as creative spaces, tools, and time for brainstorming or innovative projects, can further stimulate and harness employee creativity for enhanced job performance [27].

While there is an ample research on social media’s impact on job performance, fewer studies have explained the mediating effects of transactive memory capability and employee creativity. This multi-faceted approach remains underexplored. Existing studies focused on specific industries or regions, leaving a gap in understanding how these variables interact in generalized way. There is also a gap in integrating relevant theoretical frameworks such as social exchange theory, cognitive load theory, and creativity theories to understand the relation between social media usage, TMC, and employee creativity in enhancing job performance. Kaplan and Haenlein [28] discuss how social media can influence organizational life, including communication and performance. However, the specific mediating roles of transactive memory capability and employee creativity are not addressed. Lewis and Herndon [29] provide an overview of TMC and their relevance in team performance, and this work sets a foundation for exploring how these systems mediate this relation. Amabile [30] outlines the componential theory of creativity, highlighting factors that can enhance or inhibit creativity in the workplace. This framework can be applied to examine how social media might foster an environment conducive to creativity. However, there are limited comprehensive studies examining how social media usage translates into enhanced job performance. By addressing these gaps and building on existing literature, the proposed study offers valuable insights into how social media can enhance job performance through the mediating effects of TMC and employee creativity. The study extends existing theories on media richness, transactive memory systems, and creativity by integrating these constructs into a unified model, advancing theoretical understanding.

To study the interplay between TMC, social media usage, employee creativity, and job performance in China holds several compelling reasons. China’s unique cultural and organizational context may influence the dynamics of these variables. Understanding how TMC, social media, and creativity impact job performance in a collectivist society like China can provide insights into culturally sensitive approaches to optimize workplace efficiency. China’s position as a global economic powerhouse makes it crucial to explore factors that contribute to enhanced job performance [28]. Identifying how TMC, social media, and creativity influence performance can aid Chinese organizations in maximizing productivity and competitiveness. China is a leader in technology adoption, with a massive user base for social media platforms and innovative approaches to technology integration [16]. Studying the role of social media in fostering TMC and employee creativity can provide valuable lessons for other societies undergoing similar technological transformations. Enhancing job performance is crucial for individual career development and organizational success [12]. Investigating how TMC and creativity, facilitated by social media, contribute to job performance can offer strategies for talent development and employee engagement in the Chinese workforce [29]. Chinese companies are increasingly embracing novel organizational practices. Understanding how TMC, social media, and creativity intersect with job performance can guide these companies in structuring teams, fostering collaboration, and leveraging technology for optimal outcomes. Earlier literature little focused the empirical estimated role of TMC, social media usage and employee creativity for job performance in China. This study is intended to fill this gap by collecting the data from Chinese firms then structural equation model is applied for empirical analysis.

## 2. Conceptual framework and hypothesis

### 2.1. Theoretical foundations

Social media is an important way of modern communication, revolutionizing the way individuals interact and collaborate. In organizational context, social media platforms offer unique opportunities to enhance job performance by fostering creativity, and improving communication. This study explores the theoretical foundations underlying the role of social media in improving job performance, with a specific focus on the mediating roles of Transactive Memory Capability and employee creativity. “Media Richness Theory (MRT) provides a theoretical framework for understanding how different communication channels affect the richness of information exchange and, consequently, organizational performance. According to MRT, communication channels vary in their ability to convey complex information and provide immediate feedback” [31]. Social media, with its multimedia capabilities and real-time interactions, is considered a rich communication channel. Social media enables rapid dissemination of information across organizational boundaries, facilitating knowledge sharing and collaboration among employees. Through features like video conferencing, instant messaging, and discussion forums, social media allows for rich, interactive communication that can enhance understanding and decision-making.

“Transactive Memory Systems (TMS) Theory posits that groups develop a shared system for encoding, storing, and retrieving knowledge, with each member specializing in different domains” [32]. TMS enhances collective intelligence and problem-solving by distributing knowledge across group members. Social media serves as a source for distributing knowledge within teams, enabling members to access expertise and information from others. By facilitating the organization of knowledge through tagging, categorization, and search functionalities, social media enhances the efficiency of TMS. “Social Cognitive Theory (SCT) emphasizes the role of observational learning and social interaction in shaping individual behavior. According to SCT, individuals learn from observing others and are influenced by the social context in which they operate” [33]. Social media provides opportunities for individuals to observe and learn from others’ behaviors, including innovative practices and problem-solving strategies. Through social media, individuals are affected by norms, expectations, and feedback, which can impact their creativity and performance. In conclusion, the theoretical foundations discussed highlight the multifaceted ways in which social media can influence job performance. By providing rich communication channels, enhancing Transactive Memory Capability, stimulating creativity, and shaping social behaviors, social media significantly enhances job performance. Understanding these theoretical underpinnings can inform organizational strategies for effectively leveraging social media to improve job performance and foster innovation in the workplace.

### 2.2. Social media usage and job performance

MRT explains that the effectiveness of communication is influenced by richness of media used. Social media platforms are considered rich communication channels because they support real-time interactions, multimedia content, and immediate feedback. This richness can enhance the efficiency and effectiveness of communication within organizations, leading to better job performance [34]. Social capital theory is of view that social media facilitates the creativity and maintenance of social capital by enabling individuals to build and maintain relationships, access resources, and gain social support. Increased social capital can provide employees with valuable information, advice, and support, which can enhance their job performance [35]. By facilitating the exchange of ideas, best practices, and expertise, social media can enhance employees’ knowledge base and problem-solving capabilities, leading to improved job performance [36]. Engaged employees are more likely to perform well in their jobs. Social media increases the engagement of employees by providing platforms for social interaction, recognition, and feedback. Engaged employees are more motivated, satisfied, and committed to their work, which can positively impact their job performance.

Studies show that social media usage in organizations has positive relation with various aspects of job performance, including productivity, innovation, and collaboration [16, 37, 38]. These studies provide empirical support for positive relation between social media and job performance. Many organizations have successfully integrated social media into their workflows to improve communications and collaborations. Case studies and industry reports often highlight the positive relation between job performance and usage of social media such as project completion rates, customer satisfaction, and employee productivity [39]. It is argued that increased usage of social media platforms for work-related purposes will be associated with higher levels of job performance among employees. The underlying mechanisms for this relationship include improved communication, enhanced knowledge sharing, increased social capital, and higher employee engagement. Based on the rationale and empirical evidences, the hypothesis is formulated as follows:

*H1*: Social media usage positively affects the job performance.

### 2.3. Job performance and transactive memory capability

This relation is rooted in the idea that an organization or a team functions more effectively when its members collectively possess and utilize a shared understanding [30]. TMC suggests that individuals within a group or organization develop expertise in specific domains [22]. This specialization allows each member to become proficient in certain areas, knowing where to find information and who holds particular expertise within the group [31]. When individuals recognize and trust each other’s specialized knowledge, they can effectively coordinate their efforts. This coordination leads to efficient teamwork, reduced duplication of efforts, and smoother task execution [40]. TMC emphasizes not only the possession of knowledge but also the accessibility and retrieval of that knowledge when needed. A group with high TMC can efficiently access and utilize relevant information, leading to quicker and more accurate decision-making [33, 41]. Teams with collective knowledge sharing can synthesize diverse perspectives, leading to innovative solutions that draw upon the collective knowledge of the team [34, 42]. As the environment changes or new challenges arise, the shared understanding allows the team to quickly adapt and respond effectively to novel situations. Theoretical frameworks propose that higher levels of TMC within teams or organizations positively correlate with improved job performance [35]. This correlation occurs because TMC facilitates the efficient use of available knowledge resources, leading to enhanced task execution, problem-solving, decision-making, and innovation [11, 43]. Furthermore, TMC can indirectly influence job performance by fostering a conducive environment for creativity, collaboration, and continuous learning among team members, which are all crucial factors contributing to overall job performance [26, 44]. Overall, the theoretical relation between TMC and job performance suggests that a well-developed TMC within a group or organization contributes positively to achieving superior performance outcomes.

*H2*: *TMC has positive relationship with job performance*.

### 2.4. Employee creativity and job performance

The theoretical relation between employee creativity and job performance is based on the idea that creative thinking and innovative behaviors positively influence various aspects of job performance [45, 46]. Creative employees are adept at generating novel ideas and solutions to problems. Their ability to think outside conventional boundaries enables them to tackle challenges in unconventional ways, leading to more effective problem-solving and fostering innovation within the organization [47]. Creative individuals tend to be more adaptable to changing circumstances. They can pivot, adjust, and embrace new ideas or methods, contributing to increased flexibility within the workplace [48]. This adaptability is crucial for maintaining high job performance in dynamic and evolving environments. Employees who demonstrate creativity often produce work of higher quality. Their ability to generate innovative ideas and approaches leads to improved processes, products, or services, which positively impacts the overall quality of work output [49]. Creative individuals are inclined to take initiative and exhibit proactive behaviors. They seek out new opportunities, propose improvements, and take risks that contribute positively to achieving organizational goals and driving performance. Creative individuals often excel in collaborative settings [35]. Their openness to new ideas, ability to inspire others, and willingness to explore different perspectives can enhance team dynamics, leading to improved collective performance. Employees who have the opportunity to express their creativity tend to experience higher job satisfaction and engagement [50]. This heightened engagement translates into increased motivation, commitment, and overall job performance. The Componential Theory of Creativity and Social Cognitive Theory, suggest that creativity positively influences job performance by enhancing problem-solving abilities, fostering innovation, promoting proactive behaviors, and contributing to a more positive work environment [51]. It’s important to note that while there’s a theoretical link between employee creativity and job performance, the nature and extent of this relationship can vary across different organizational contexts, roles, and industries [28]. However, fostering a culture that encourages and supports creativity can significantly contribute to enhancing overall job performance within an organization.

*H3*: *Employee creativity increase the job performance of individuals*.

### 2.5. Mediating role of transactive memory capability(TMC)

Social media platforms are sources of exchange and dissemination of information. Theoretically, social media can enhance TMC, creating a collective understanding of who possesses specific knowledge within a team or organization [52]. Social media usage may influence TMC by enabling and enhancing the sharing and retention of knowledge. As individuals engage with social media tools, they may develop a collective awareness of each other’s expertise and thereby contribute to the development of TMC within teams or organizations [13]. Social media usage helps build and maintain TMC by facilitating communication, collaboration, and information sharing among employees. This strengthens the collective memory system within the organization. A robust TMC enhances job performance by enabling efficient task allocation, improved problem-solving, and better coordination. Employees can leverage the collective expertise of their colleagues, leading to higher performance outcomes. The theoretical framework suggests that social media influences job performance not only directly but also indirectly through its effects on TMC [29]. It posits that usage of social media platforms contributes to the development of TMC, influencing job performance [53]. Empirical research exploring this theoretical framework investigates how social media usage patterns within organizations affect the development of TMC, how they influence job performance [54].

*H4*: *TMC mediates the relation of social media use and job performance*.

### 2.6. Mediating role of employee creativity

The exposure to diverse perspectives and collaborative opportunities provided by social media can stimulate creative thinking and problem-solving. The mediating role of employee creativity suggests that social media usage impacts job performance through its influence on creativity. Employees who use social media may develop higher creativity levels, which in turn, positively affects their job performance [55]. Social media allow to access a wealth of information and share knowledge quickly and easily. This constant exposure to new ideas and diverse perspectives can spark creative thinking. Employees can connect with colleagues, industry experts, and thought leaders, because social media provides tools and spaces for brainstorming and idea sharing. Platforms like discussion forums, professional networks, and collaborative tools can stimulate creative processes by allowing employees to discuss and refine ideas collaboratively [21]. As employees engage with social media, they gain access to diverse information and collaborative opportunities. This engagement enhances their creativity by providing new ideas and perspectives. The enhanced creativity resulting from social media engagement enables employees to approach their work more innovatively and efficiently [56]. This creative approach positively impacts their job performance. Social media acts as a catalyst for creativity by providing access to diverse information and collaborative opportunities. This enhanced creativity improves the job performance through innovative problem-solving, adaptability, and increased efficiency. Understanding this mediation process can help organizations leverage social media and foster creativity to boost overall job performance.

*H5*: *Employee creativity mediates the relationship of social media usage and job performance*.

On the basis of above discussion, the conceptual framework of this study is given in the following Fig 1.

**Fig 1:** Conceptual framework.

“Social Exchange Theory (SET) can serve as an overarching theoretical foundation for this study. SET posits that social behavior is the result of an exchange process where individuals seek to maximize benefits and minimize costs. This theory is relevant for understanding how social media usage impacts TMC and employee creativity, which in turn affects job performance. Social media platforms facilitate interactions and exchanges among employees, enabling them to share information, knowledge, and expertise” [28]. These exchanges are mutually beneficial, as employees gain access to valuable resources that enhance their capabilities. Through consistent interactions on social media, employees build trust and reciprocity, essential elements of SET. Trust and reciprocity help in the development of TMC as employees rely on each other for information and expertise. Employees utilize the enhanced TMC and creativity developed through social media exchanges to improve their job performance. The benefits of efficient task allocation, innovative solutions, and effective collaboration are realized in better performance outcomes [57]. The reduced effort required to find information and the improved efficiency in task completion as a result of TMC and creativity help minimize the costs associated with job performance. By grounding the proposed model in Social Exchange Theory, the study can effectively explain how social media usage leads to enhanced job performance through the mediating roles of TMC and employee creativity. This theoretical foundation provides a robust framework for understanding the dynamics of social interactions and exchanges that drive the relationships in the proposed model.

## 3. Materials and methods

The “Research Ethics Committee” of the Xinyang Agriculture and Forestry University approved the study vide no. XAFU/2023/153 on January 6, 2023. The data is collected from March 1, 2023 to June 30, 2023. The participants gave a written consent to participate in the study so online resources are used to send the questionnaire. The study considers the employees from various hierarchical levels, including entry-level workers, middle management, and senior management, to capture a comprehensive view of social media usage. The participants were employees from different departments and job functions, like marketing, human resources, research and development, sales, and customer service. Data was collected using an online questionnaire. The sample for the study was selected from the larger population using a convenient sampling technique. “Convenience sampling is a non-probability sampling technique where subjects are selected because of their convenient accessibility and proximity to the researcher. This method is often used in exploratory research where the aim is to get a quick, approximate understanding of a phenomenon rather than achieving a statistically representative sample of the entire population” [58]. Participants are chosen based on their availability and willingness to take part in the study. This can include individuals who are easy to reach or who volunteer to participate. Since it involves selecting participants who are readily available, it tends to be less expensive and quicker to administer compared to other sampling methods. Convenience sampling is a practical and cost-effective method for gathering initial data or conducting exploratory research [59–61]. For studies aiming for rigorous, generalizable results, more systematic sampling methods are preferred.

The 5-point Likert scale is used to measure the constructs and items of questionnaire. Employees having the age of more than 18 years are selected for this study. We sent 1090 questionnaires and 816 questionnaires were selected for further empirical analysis. The incomplete and ambiguous questionnaires were excluded from the analysis. Based on the earlier literature, the study used the age, gender, education, and residence are used as control variables in the study. The study used AMOS for empirical analysis as the decision to utilize AMOS for conducting Structural Equation Modeling (SEM) in this study was based on several factors that make AMOS a preferred choice over other software packages. AMOS is specifically designed for SEM, offering a user-friendly interface and robust features that are well-suited for analyzing complex relationships among variables. Its interface is tailored to SEM workflows, offering intuitive tools for model specification, estimation, and evaluation. “AMOS offers a variety of fit indices to assess the goodness of fit of SEM models, such as the Comparative Fit Index (CFI), Tucker-Lewis Index (TLI), and Root Mean Square Error of Approximation (RMSEA)” [58–61]. These indices help researchers evaluate the overall fit of the model to the data. AMOS also includes advanced features for testing mediation, moderation, and multiple group analyses, which are relevant to the objectives of this study. The descriptive analysis is given in Table 1.

**Table 1:** Descriptive analysis (N = 816).

Category	Item	Frequencies	Percentage
Gender	Male	409	50.12
	Female	407	49.88
Age	18–28 Years	297	36.40
	29–39 Years	316	38.73
	40 and above	203	24.88
Qualification	High School	44	5.39
	Bachelor	461	56.50
	Master and above	311	38.11
Residence Area	Urban	452	55.39
	Rural	364	44.61

The Table 1 is outlining the demographic information of respondents. The study’s respondents were diverse in terms of gender, with a relatively equal distribution between male and female participants. This gender balance ensures that the study’s findings are representative and applicable to both male and female employees. The age range of respondents varied, with a significant proportion falling in the 29–39 age group. This suggests that the study’s findings may be more relevant to younger employees, who are often more adept at using social media and may exhibit higher levels of creativity. The majority had a bachelor’s degree, suggesting that findings may be more applicable to knowledge workers. Moreover, majority of the respondents in the sample belongs to urban areas.

### Common method bias

Harman’s single-factor test is a preliminary method to check the common method bias (CMB). “This test involves conducting an exploratory factor analysis on all items of your study and examining the unrotated factor solution. If the first factor accounts for more than 50% of the total variance, this suggests a significant presence of common method bias but if the first factor does not account for the majority of the variance, it suggests that common method bias is less likely to be a problem in your data. In this case, the first factor accounts for 32% of the total variance, which is below the 50% threshold” [62, 63]. This suggests that common method bias might not be a significant concern in your study.

### Estimated results

The estimated results of validity and reliability of constructs are shown in Table 2.

**Table 2:** Reliability and validity test.

Variables	Item	Loadings	CR	CA	KMO	Barlett’s test		
						χ^2^	df	Sig
Social Media Usage (SOUG)	SOUG1	0.79	0.84	0.83	0.80	746	5	0.00
	SOUG2	0.72						
	SOUG3	0.81						
	SOUG4	0.77						
	SOUG5	0.81						
Transactive Memory Capability (TRMC)	TRMC1	0.66	0.82	0.81	0.77	637	4	0.01
	TRMC2	0.69						
	TRMC3	0.72						
	TRMC4	0.85						
	TRMC5	0.86						
Job Performance (JPRF)	JPRF1	0.82	0.87	0.82	0.77	613	4	0.01
	JPRF2	0.81						
	JPRF3	0.73						
	JPRF4	0.79						
	JPRF5	0.77						
Employee Creativity (ELCT)	ELCT1	0.72	0.85	0.79	0.75	412	5	0.00
	ELCT2	0.79						
	ELCT3	0.81						
	ELCT4	0.88						
	ELCT5	0.79						

Note: “CR = Construct reliability; CA = Cronbach’s alpha; KMO = Kaiser–Meyer–Olkin; AVE = Average variance extracted”

“The values of CA of all variables are above than 0.7 indicate internal consistency. The convergent validity is measured through CR, Barlett’s test, and KMO values” [64]. The results show that all values of CR are greater that threshold level of 0.8, while value of KMO is greater than 0.7, and Bartlett’s test is also significant. Pearson’s correlation coefficient is applied and findings of discriminant validity are reported in Table 3.

**Table 3:** Discriminant validity.

	SOUG	TRMC	JPRF	ELCT
**SOUG**	0.88			
**TRMC**	0.45	0.85		
**JPRF**	0.62	0.63	0.86	
**ELCT**	-0.51	-0.42	-0.59	0.85

Note: “All values are significant at 1% while diagonal value is square root of AVE”.

“The values of correlation coefficients are smaller than square root of AVE depicting that internal correlations between the observed variables are higher than external correlations” [63–65], so discriminatory validity exists.

### Structural equation modeling

SEM method is used to investigate the effect of SOUG on JPRF and TRMC. The results are shown in Table 4.

**Table 4:** Structural parameter estimate.

Hypotheses	Standardized Path Coefficient	t-value	Result
SOUG→ JPRF	0.537*	7.564	Yes
TRMC →JPRF	0.413*	6.276	Yes
ELCT→ JPRF	0.516*	8.362	Yes
SOUG →TRMC→ JPRF	0.452*	6.382	Yes
SOUG→ ELCT→ JPRF	0.516*	8.527	Yes
x^2^/df = 2.989* RFI = 0.910	NFI = 0.901 GFI = 0.912	RMSEA = 0.071 IFI = 0.924	CFI = 0.910 RMR = 0.059

Note: “* shows significance at 1%”.

The results depict that all path coefficients are significant and positive so hypotheses are confirmed. “The (x^2^/df) ratio was below 5, and the RMR score was 0.063, while the RMSEA score was 0.079, both below the acceptable threshold of 0.08. Additionally, the GFI, CFI, RFI, NFI, and IFI values were all greater than the recommended values of 0.90” [58, 59].

The mediation analyses are shown in Table 5. The empirical results reveal that transactive memory capability and creativity of employees, partially mediate the relationship.

**Table 5:** Mediation effect.

Effect of SOUG on TRMC	Effect of TRMC on JPRF	Direct Effect	Indirect Effect	Confidence Interval		P-value	Result
				L Bound	U Bound		
0.33	0.38	0.43**	0.14**	0.074	0.151	0.001	Partial
Effect of SOUG on ELCT	Effect of SOUG on JPRF						
0.32	0.36	0.42**	0.15**	0.071	0.183	0.002	Partial

Note: ** show significance at 5%.

## 4. Discussion

This study investigated the impact of SOUG on TRMC and how TRMC influences the JPRF. The first hypothesis reveals that social media usage improves the job performance. The findings of the study are supported theoretically and empirically. Media Richness Theory posits that communication effectiveness depends on the richness of the media used. Rich media can convey more information and provide immediate feedback, which enhances communication efficiency [66]. Social media platforms are considered rich media as they support multimedia content, real-time interactions, and immediate feedback. In China, platforms like WeChat and Weibo facilitate rich interactions among employees, enhancing communication and collaboration, which in turn improves job performance [67]. Social capital theory suggests that social networks provide value through the relationships and resources accessible within those networks. In China, social media enhances social capital by enabling employees to build and maintain professional relationships, access valuable information, and gain support from their networks. This increased social capital can lead to better access to resources and information, thereby improving job performance [68]. “Knowledge management theory focuses on the processes of creating, sharing, and applying knowledge within organizations to improve performance” [69]. Social media platforms in China facilitate knowledge sharing by providing spaces for discussion, document sharing, and collaborative problem-solving. This enhances the overall knowledge base of employees, leading to more informed decision-making and improved job performance. The earlier literature [22, 37, 70] found that social media usage in Chinese firms significantly improved internal communication and collaboration among employees, leading to enhanced job performance. The study highlighted that platforms like WeChat allowed for real-time updates and collaborative project management, improving efficiency and output. It is explored how social media usage influenced job performance in Chinese companies. The study found that employees who actively used social media for professional networking had greater access to resources and support, which enhanced their job performance. The increased social capital facilitated by social media enabled employees to leverage their networks for information and assistance [47]. Tencent, a leading Chinese technology company, effectively uses social media platforms and company reports that social media integration has streamlined project management, improved team coordination, and increased overall productivity, demonstrating the positive impact on job performance.

The results also support Hypothesis 2, postulating a positive relation between TRMC and JPRF. “Transactive memory theory posits that groups develop a shared system for encoding, storing, and retrieving information” [16]. Each member specializes in different domains of knowledge, and the collective memory is greater than the sum of individual memories. A well-developed TRMC within an organization allows employees to access and utilize the expertise of their colleagues efficiently. This leads to improved decision-making, problem-solving, and innovation, enhancing overall job performance. Resource-Based view theory suggests “that organizations can achieve competitive advantage by developing and utilizing unique resources and capabilities” [48]. Social Exchange Theory emphasizes the importance of reciprocal relationships and the exchange of resources (including knowledge) within social networks. TRMC fosters a culture of knowledge sharing and collaboration, where employees are more likely to share their expertise and rely on others’ knowledge. This reciprocal exchange of information enhances job performance through improved efficiency and innovation [19]. By distributing cognitive tasks and knowledge across the team, TRMC reduces individual cognitive load. Employees can focus on their areas of expertise while relying on others for additional information, leading to better performance outcomes.

A study Liang et al. [34] found that teams with well-developed TRMC performed better on complex problem-solving tasks. In the context of China, research by Wang et al. [57] demonstrated that TRMC in Chinese firms led to more effective decision-making and quicker problem resolution, directly improving job performance. Research by Zhang et al. [71] in Chinese organizations showed that TRMC facilitated better collaboration among team members. The study found that teams with strong TRMC were more innovative, as they could combine their diverse knowledge to generate creative solutions, enhancing job performance. A study [33] for the Chinese manufacturing sector indicated that TRMC enabled more effective knowledge integration and utilization. Teams with robust TRMC were able to harness and apply their collective knowledge more efficiently, leading to improved job performance metrics such as productivity and quality. Research [14] found that TRMC positively impacted employee satisfaction and retention in Chinese firms. Employees who felt their knowledge was valued and utilized within the TRMC were more satisfied with their jobs, leading to higher engagement and better performance. Huawei, a leading Chinese technology company, has implemented TRMC practices to manage its extensive knowledge base. By fostering specialized knowledge areas and encouraging knowledge sharing, Huawei has improved its R&D efficiency and innovation capacity, leading to better overall job performance.

The study outcomes validate Hypothesis 3, describing that employee creativity improves the job performance. The findings are supported by theoretical and empirical evidences. Amabile’s componential theory of creativity theory explains “that creativity arises from the interaction of three key components: domain-relevant skills, creativity-relevant processes, and intrinsic task motivation” [30]. In the workplace, employees who possess these components can generate novel and useful ideas, leading to innovative solutions and improvements in processes, products, or services. This creativity directly contributes to enhanced job performance by enabling organizations to adapt and compete effectively. Creativity is viewed as a valuable resource that leads to develop the new services, products, and processes. Organizations that nurture and leverage employee creativity can differentiate themselves from competitors and improve overall performance [39]. Job characteristics model asserts that job design influences employee motivation, satisfaction, and performance. Key job characteristics include task significance, autonomy, and feedback [53]. Jobs that are designed to be challenging and provide autonomy encourage employees to engage in creative thinking. When employees feel their work is meaningful and they have the freedom to explore new ideas, their creativity enhances their job performance [61]. Social exchange theory explains the reciprocal nature of relationships and exchange of resources, including knowledge and support. In supportive work environments, employees are more likely to share creative ideas. Positive social exchanges foster a culture of trust and collaboration, which can enhance creativity and, in turn, job performance.

A study [44] in Chinese firms found that employee creativity significantly contributed to innovative outcomes. Creative employees were better at solving complex problems and generating novel ideas, leading to improved job performance and organizational innovation. Research [63] indicated that employee creativity was positively correlated with productivity in Chinese manufacturing firms. The study demonstrated that creative employees could streamline processes and introduce efficiency improvements, enhancing overall job performance. A study [10] for the Chinese service industry found that employee creativity led to higher levels of customer satisfaction. Creative employees were able to tailor services and create unique customer experiences, resulting in better job performance metrics related to customer feedback and retention. Research highlighted that employee creativity contributed to organizational adaptability in Chinese technology firms. Creative employees helped organizations respond more effectively to market changes and technological advancements, leading to sustained job performance improvements [52]. Alibaba, one of China’s leading e-commerce companies, emphasizes creativity and innovation among its employees. The company fosters a creative culture through initiatives like internal hackathons and innovation labs. This focus on creativity has resulted in continuous improvements in their platform, customer experience, and overall job performance.

The hypothesis 4 confirms that TRMC mediates the relation between SOUG and JPRF by enhancing how employees use social media to develop, store, and retrieve knowledge, improving their performance. The mediation process involves social media usage positively influencing the development and functioning of TRMC, which then leads to better job performance [21]. Social media facilitates the sharing of knowledge and information among employees, helping them identify who holds specific expertise within the organization. Through social media interactions, employees can build and strengthen networks of expertise, knowing who to turn to for specific information or skills [45]. TRMC allows employees to quickly access the right information from the right people, leading to more efficient problem-solving and decision-making. By relying on the expertise of their colleagues, employees can collaborate more effectively, leading to improved task performance [62]. TRMC reduces the cognitive load on individual employees by distributing the responsibility for storing and retrieving information across the team. Employees who actively use the social media for work purpose may experience a direct positive impact on their job performance due to improved communication and access to information. Social media usage enhances the development and functioning of TRMC by facilitating knowledge sharing, building expertise networks, and improving communication and coordination [28]. A well-functioning TRMC leads to better job performance as employees can efficiently retrieve and apply knowledge, collaborate effectively, and reduce cognitive load. Through these interactions, the employee develops a strong network of expertise, knowing who has the relevant knowledge for various tasks. The employee can quickly access the needed information from the right colleagues, leading to efficient problem-solving, effective collaboration, and higher productivity [47]. Research supports the notion that social media usage can enhance TRMC, which in turn positively impacts job performance. The study [22] found that SOUG within organizations facilitates the development of TRMC by improving the visibility of expertise and enhancing knowledge sharing. Another study [58] demonstrated that TRMC mediates the relation between knowledge-sharing behaviors and team performance, highlighting the importance of TRMC in translating social media usage into performance gains.

The hypothesis 5 reveals that employee creativity mediates the relation between SOUG and JPRF. The mediation process involves SOUG positively influencing employee creativity, which lead to better JPRF. Social media provides access to a vast amount of information and knowledge from diverse sources. Employees can leverage this information to generate new ideas and innovative solutions [67]. Moreover, **s**ocial media facilitates collaboration and networking with colleagues, experts, and communities. This interaction can spark creativity by exposing employees to different perspectives and feedback. Exposure to innovative content, trends, and best practices on social media can inspire employees to think creatively and apply new approaches to their work. Creative employees are better equipped to develop innovative solutions to work-related problems, leading to improved efficiency and effectiveness [18]. Employees who actively use social media for work purpose may experience a direct positive impact on their job performance due to improved communication and access to information. Increased creativity leads to better job performance as employees apply their creative skills to solve problems, improve processes, and innovate in their roles. The total effect of SOUG on JPRF includes both direct and indirect effect mediated by employee creativity. Research supports the notion that SOUG can enhance employee creativity, which in turn positively impacts job performance. The study [44] found that SOUG for professional purpose enhances creativity by facilitating knowledge sharing and collaborative learning. By leveraging social media effectively, organizations can foster a creative work environment that leads to superior job performance.

### 4.1. Limitations

There are some limitations as the study employed cross-sectional data while longitudinal studies are needed to establish causal relationships. The sample may not be representative of all organizational contexts or industries. The findings might not be generalizable to organizations with different cultures, structures, or levels of social media adoption. Future research should consider diverse samples across various sectors and geographic regions. Acknowledging these limitations is crucial for interpreting the study’s findings and understanding their implications. Future research should address these limitations by employing longitudinal designs, using objective measures, diversifying samples, and considering additional contextual and control variables. By doing so, researchers can build on the current study’s insights and further elucidate the role of social media in enhancing job performance through TRMC and employee creativity.

## 5. Conclusions

Due to prevailing increase in popularity of social media, organizations are using these platforms to increase the mutual collaborations among team members while research on this topic is limited. This study provided valuable insights explaining the mechanisms through which SOUG can enhance employee performance in organizational settings. By exploring the mediating roles of TRMC and employee creativity, the study offers a nuanced understanding of how social media can be leveraged to improve job performance. Social media usage improves the job performance of employees through better communications, fostering the knowledge sharing, and collaboration among employees. While TRMC significantly mediates the relation between SOUG and JPRF. Social media helps to build and enhance TRMC by enabling employees to identify, store, and retrieve knowledge efficiently, leading to improved problem-solving, collaboration, and overall job performance. Employee creativity also has a crucial mediating role in relation between SOUG and JPRF. Social media provides a platform for employees to access diverse information and engage in collaborative interactions, fostering creativity. This creativity, in turn, translates into innovative solutions and improved job performance.

### 5.1. Implications

#### 5.1.1. Theoretical implications

The study extends existing theoretical frameworks in organizational behavior, information systems, and knowledge management by elucidating the mechanisms through which social media usage impacts job performance. The findings offer several theoretical contributions. The study demonstrates that social media not only provides rich communication channels but also enhances cognitive and creative processes within organizations. It extends Media Richness Theory by highlighting the multifaceted roles of social media in facilitating knowledge sharing and fostering innovation. The study also contributes to TRMC Theory by showing how SOUG strengthens the development and functionality of TRMC. It provides empirical evidence that social media serves as a critical tool for building and maintaining a collective memory system, thus supporting efficient knowledge retrieval and application. The study is also addition in understanding of creativity theories by positioning employee creativity as a mediator between SOUG and JPRF. By integrating theories from media richness, transactive memory systems, creativity, job performance, and the knowledge-based view of the firm, the research offers a holistic understanding of the mechanisms through which social media can enhance job performance. These contributions not only advance academic knowledge but also provide a foundation for future research to further explore the complex relationships between social media usage, cognitive and creative processes, and organizational outcomes.

#### 5.1.2. Practical implications

The study also offers several practical implications for organizations aiming to enhance job performance through effective social media usage. By understanding the mediating roles of Transactive Memory Capability and employee creativity, managers can develop strategies to leverage social media as a powerful tool for improving workplace productivity and innovation. Organizations should encourage the use of social media platforms for knowledge sharing. Creating groups or communities on platforms like Slack, Microsoft Teams, or enterprise social networks can help employees share expertise and information efficiently. Implement tools to map and identify areas of expertise within the organization. Social media profiles and interactions can help build a comprehensive understanding of who knows what, aiding in quicker problem-solving and decision-making. Provide training programs to educate employees on the effective use of social media for professional purposes. Training should focus on how to leverage social media for networking, knowledge sharing, and collaboration. Conduct workshops that focus on enhancing creative thinking and problem-solving skills, showing employees how to use social media as a source of inspiration and innovation. Foster a culture that encourages open communication and collaboration through social media. Regular virtual brainstorming sessions, innovation contests, and collaborative projects can stimulate creativity. Implement recognition and reward systems for employees who contribute creative ideas and solutions, highlighting the role of social media in these achievements. Ensure employees have access to the necessary social media tools and platforms that facilitate creativity and innovation. Invest in technologies that support collaborative work environments. Encourage leaders to actively participate in social media interactions, demonstrating the importance of these platforms for innovation and performance. Develop integrated social media strategies that align with the organization’s goals and objectives. Ensure that social media usage is directed towards achieving performance improvements and fostering innovation. The practical implications of this study highlight the importance of strategically leveraging social media to enhance job performance through improved Transactive Memory Capability and employee creativity. By implementing these strategies, organizations can create a more collaborative, innovative, and efficient work environment, leading to sustainable competitive advantage and superior performance outcomes.

## Supporting information

S1 File (DOCX)

S1 Data (XLSX)
